The article "Effects of Panax notoginseng saponins on severe acute pancreatitis through the regulation of mTOR/Akt and caspase-3 signaling pathway by upregulating miR-181b expression in rats" was retracted in 2022. Reasons: duplicated images; unreliable data; concerns about the images.

# Effects of Panax notoginseng saponins on severe acute pancreatitis through the regulation of mTOR/Akt and caspase-3 signaling pathway by upregulating miR-181b expression in rats

**DOI:** 10.1186/s12906-018-2118-8

**Published:** 2018-02-05

**Authors:** Ming-wei Liu, Rui Wei, Mei-xian Su, Hui Li, Tian-wen Fang, Wei Zhang

**Affiliations:** 1 Department of Emergency, the First Hospital Affiliated To Kunming Medical University, 295 Xichang Road, Wu Hua District, Kunming, 650032 China; 2 Intensive Care Unit, The Second Hospital Affiliated To Kunming Medical University, 1 Mayuan Road, Wu Hua District, Kunming, 650106 China; 3 Department of Postgraduate, Kunming Medical University, 1168, Chunrong West Road, Chenggong District, Kunming, 650500 China

**Keywords:** Acute pancreatitis, *Panax notoginseng saponins*, miR-181b, Taurocholate, Rat

## Abstract

**Background:**

In China, *Panax notoginseng* has been used to treat oxidative stress-related diseases for a long time. *Panax notoginseng saponins* is an extract from *Panax notoginseng Ledeb*. Its therapeutic potential is related to antioxidant activity, but related mechanisms are still unclear. The study aims to assess the protection effects of *Panax notoginseng saponins* in the taurocholate-induced rat model of acute pancreatitis (AP) and explore underlying mechanisms.

**Methods:**

A rat model of severe acute pancreatitis (SAP) was established in rats induced with taurocholate. *Panax notoginseng saponins* was firstly administered in the treatment group via intravenous injection. After 2 h, taurocholate administration was performed. After 24 h, the expression levels of miR-181b, Beclin1, LC3-II, Akt and mTOR from pancreas tissues were measured by Western Blotting and RT-PCR. Then the expression levels of Caspase-3 and Blc-2 were determined by immunohistochemistry. Apoptosis was assessed by the TUNEL assay. Amylase and lipase in serum were determined by ELISA and pancreatic water contents in pancreatic tissue were measured. After eosin and hematoxylin staining, the histologic analysis was performed.

**Results:**

After SAP induction by taurocholate and the treatment with *Panax notoginseng saponins* for 24 h, we detected the up-regulated miR-181b, the reduced Bcl-2 expression, the increased activity of mTOR/Akt, the blocked Beclin1 and LC3-II expressions, and the enhanced Caspase-3 expression. Serum lipase and amylase levels were significantly decreased in the treatment group of *Panax notoginseng saponins* compared to the control group. Histological analysis results verified the attenuation effects of *Panax notoginseng saponins* on taurocholate-induced pancreas injury, apoptosis, and autophagy.

**Conclusion:**

By up-regulating the miR-181b expression level, *Panax notoginseng saponins* significantly reduced taurocholate-induced pancreas injury and autophagy and increased apoptosis. The significant protection effects of *Panax notoginseng saponins* suggested its potential in treating taurocholate induced-acute pancreatitis.

## Background

As an abdominal emergency, acute pancreatitis (AP) involves concomitant organ failures and other eventful complications and generally causes considerable deaths [1]. Pancreatitis is generally ascribed to the self-digestion of pancreatic acinar cells after inactive trypsinogen is activated into trypsin [1, 2]. The pancreatitis pathology of has not been completely explored. Currently, there is no effective medication for treating SAP. The main therapeutic approaches for SAP are symptomatic treatments including gastric decompression, the provision of pain relief, and the correction of fluid, electrolyte, and pH balances [3]. Many researchers are screening active ingredients from traditional Chinese medicine (TCM) to assess their potential to treat SAP.

Sanqi (*Panax notoginseng*) is a member of the Araliaceae family. In China, it has been used to treat various diseases for a long time. According to TCM theory, *Panax notoginseng* can reduce blood stasis. As one of the main active components in Sanqi. Panax notoginseng saponin (PNS) exerts the antioxidant activity, inhibits cell growth, and induces apoptosis of cancer cells [4]. PNS exerted a protection effect on oxidative stress-induced apoptosis and damage in bone marrow stromal cells [4], primary astrocytes, and a neuroblastoma cell line, SH-SY5Y [5].

Three death pathways may be evoked in the injury of acinar cells in AP: apoptosis, necrosis, and autophagy [6]. In autophagy, cytoplasmic components are delivered to autophagosome and lysosome for degradation. As the central organelle, autophagosome can decompose cytoplasmic matrix and remove intracellular pathogens. Autophagy can show devastating effects through activating trypsinogen into trypsin in the early stage of acute pancreatitis (AP). AP led to the inhibition of lysosomal degradation and autophagy processing/maturation, thus displaying a dysregulation function of autophagic flux contributing to the progression of AP [7]. Autophagic function is predominantly regulated by the Akt/mTOR kinases, and thus the mTOR/Akt autophagy pathway is a key influencing cellular process of the functions of pancreas in AP [8]. The mTOR inhibitor rapamycin is the most commonly used agent to increase autophagy [8].

Necrosis and apoptosis largely affect the development of AP [9]. In the early AP phase, several factors can lead to deaths of pancreatic acinar cells. Necrosis of acinar cells activates trypsin. However, apoptosis of acinar cells also decrease trypsin activity. Necrosis initiates inflammation, whereas apoptosis protects acinar cells [9, 10]. In vitro studies indicated that the injury/dysfunction of nonpancreatic organ in AP was mainly caused by apoptotic epithelial cell death [11] and could be enhanced by administering apoptosis inducers. In order to alleviate AP, it is necessary to select the target of pancreatic tissues rather than nonpancreatic tissues [12].

In apoptotic cells, caspase-3 is activated by intrinsic (mitochondrial) and extrinsic (death ligand) pathways [13, 14]. Caspase-3 zymogen cannot show the activity until it is cleaved after apoptotic signaling events [15]. Bcl-2 is a key anti-apoptotic protein.

As the key major regulator in gene expression, miRNAs play important roles in apoptosis, stress response proliferation, development, and differentiation [16–19]. New roles of miRNAs in the regulation of autophagy were reported [20]. For the first time, Zhu et al. reported that miRNA was involved in cancer and autophagy and experimentally proved that miR-30a targeted Beclin-1 [21] and indicated that Beclin-1 was down-regulated by miR-30a. The functions of miR-30a-mediated autophagy were further demonstrated [22, 23]. By inhibiting autophagy, miR-30a can sensitize tumor cells to cisplatin [24]. Therefore, chemoresistance may be overcome by regulating autophagy via miRNA.

Other miRNAs might be involved in the autophagic process. MiR-98, miR-124, miR-130, miR-142, and miR-204, might regulate autophagy [25, 26]. The miR-181 family of miRNAs is a broadly conserved group of miRNAs and its members affect cell proliferation, differentiation and death [27, 28]. They have also been implicated in regulating autophagy [29]. However, the contribution of miRNA-181b in autophagy-related diseases, especially AP, is still unclear. Whether miR-181b functions as an autophagy and apoptosis-responsive miRNA to regulate the pancreatitis response to autophagy by regulating mTOR/Akt and apoptosis signaling pathway is still unknown.

Animal studies showed that *Panax notoginseng saponins* could protect the structure and function of various organs and decrease the incidence of complications [8, 30, 31]. However, the mechanism of *Panax notoginseng saponins* in the decrement of AP had not been fully investigated. Inhibiting autophagy and increasing apoptosis induction might be a promising approach to alleviate pancreatitis. This study aims to evaluate the functions of miR-181b signaling pathway in taurocholate-induced AP in rats. Furthermore, we also examined the effects of PNS administration on taurocholate-treated rats with AP by regulating autophagy and apoptosis. We selected the model of pancreatitis based on apoptosis and autophagy injury to acinar cells induced by hyperstimulation with clinical biliary pancreatitis sodium taurocholate. In the study, PNS treatment ameliorated sodium taurocholate-induced pancreatitis by increasing apoptosis and inhibiting autophagy, suggesting that PNS might have the application potential in the treatment of pancreatitis by regulating miR-181b expression. MiR-181b might play a significant role in AP biology and represent an interesting new therapeutic target for AP.

## Methods

### Plant materials

*Panax notoginseng* (purity of 82.50%) was purchased from Wenshan, Yunnan Province, China. Dr. Chong-Zhi Wang identified all herbal materials according to the Chinese Pharmacopoeia. Chen. Plant materials were stored in Yunnan College of Traditional Chinese Medicine.

### PNS extracts prepared from *Panax notoginseng*

To obtain PNS extracts, 500 g crude material of *Panax notoginseng* (Sanqi) was subjected to extraction and purification according to the following procedures. Crushed powder was added into 4 L of 70% (*v*/v) ethanol, and extracted twice for 2 h with refluxing. Extracts were evaporated by a rotary evaporator. PNS was purified on D101 resins and washed with 0.1% (v/v) ammonia, water, and 70% (v/v) ethanol. The fraction washed with ethanol was collected and evaporated. The residue was dried in a freezing dryer. All solution fractions were respectively diluted to 5 μg/mL (herbal weight per solution volume) with 1640 medium for analysis.

### High-performance liquid chromatography (HPLC) analysis of PNS extracts

The Waters 2960 HPLC system (Milford, MA) was used to anlyze PNS extracts. The separation was performed on an Alltech Ultrasphere C18 column (5 μm, I.D.: 250 × 3.2 mm) (Deerfield, IL) and a C18 guard column (5 μm, I.D.: 7.5 × 3.2 mm). Firstly, 20 μL of diluted sample solution was injected into the column for elution (1.0 mL/min, room temperature). Acetonitrile and water were respectively used as Solvent A and Solvent B. The gradient elution was performed in the following steps: starting with 17.5% Solvent A and 82.5% Solvent B, 21% A for 20 min, 26% A for 22 min, 36% A for 13 min, 50% A for 9 min, 95% A for 5 min, and 17.5% A for 11 min. in the analysis, the detection wavelength was 203 nm. According to the HPLC analysis results, 100 mL of PNS extracts contained 3.84 mg *Panax notoginseng* Rl, 17.25 mg ginsenoside Rgl, 18.16 mg ginsenoside Rbl, and 13.8 mg ginsenoside Rd. (Fig. 1).

**Fig. 1:** Chromatograms of samples and reference substances. **a** Chromatogram of reference substances. **b** Chromatograms of the following samples: 1, *Panax notoginseng* Rl; 2, ginsenoside Rgl; 3, ginsenoside Rd.; 4, ginsenoside Rbl

### Cell culture

AR42J cell lines from the American Type Culture Collection (ATCC) were cultured at 37 °C in DMEM composed of 5% FBS, streptomycin (100 units/mL), penicillin (100 units/mL), and amphotericin B (50 μg/L) in a humidified atmosphere containing 5% CO_2_. Then the cells were sub-cultured into 6-well plates and maintained until subconfluence.

### MiRNA mimics, inhibitors, and transfection

AR42J cells were cultured to the confluence of 40% in 6-well plates. MiR-181b mimics, MiR-181b mimic-negative control (NC), miR-181b inhibitor, or miR-181b inhibitor-NC (Invitrogen, Carlsbad, CA, USA) were mixed with Lipofectamine 2000 (Invitrogen), and then added into the culture medium. After transfection for 24 h, total RNA and proteins were extracted for qRT-PCR and western blotting.

### Tail intravenous administration of AdCMV-miR-181b

AdCMV-miR-181b was constructed as previously described [32, 33]. The constitutively active miR-181b expression construct was delivered to rats by intravenous administration of 1 × 10^9^ PFU of AdCMV-miR-181b at 10 d, at the time of taurocholate-induced pancreatitis. Control rats received empty adenoviral vector at the same time.

### Animals

Male Sprague Dawley rats were housed under pathogen-free conditions at a relative humidity of 30~ 70% in Kunming Medical University. At the beginning of the experiments, 8~ 9 weeks old rats were maintained on standard laboratory chow and water ad libitum. All the animal experiments were approved by the Ethics Committee of the Institute of Yunan University of Traditional Chinese Medicine (TCM).

### Taurocholate-induced SAP model

The rats were anaesthetized under aseptic conditions by intraperitoneal injection of 1% pentobarbital sodium (35 mg/kg body weight) (Wuhan Dinghui Chemical Co., Ltd., Wuhan, China). According to the previous method [34], SAP models were prepared. After median epigastric incision in the abdomen, hepatic hilus, the bile-pancreatic duct, common hepatic duct, and the duodenal papilla inside the duodenum duct wall were identified. A segmental epidural catheter was firstly inserted into the duodenum cavity and then into the bile-pancreatic duct along papilla. Two microvascular clamps were used to nip the two ends of the bile-pancreatic duct. Then, with a microinfusion pump, 5% sodium taurocholate was injected into the bile-pancreatic duct (0.2 mL/min, 1.5 mL/kg body weight). In 5 min, the epidural catheter and microvascular clamp were removed. The abdomen was closed until active bleeding was not observed in the abdominal cavity.

### Animal groups and treatments

Sixty rats were divided into the following 3 groups in a random manner: the SAP model group (model group), the Sham operation group (SO group), and the PNS group (treatment group) and each group contained 20 rats. Before the surgery, the rats of the treatment group were injected with PNS extracts (50 mg/kg) by intravenous injection administration every 8 h. The rats of the SO and SAP model groups were injected with the same volume of saline. The rats in each group were anesthetized with 1% pentobarbital sodium (35 mg/kg body weight, Wuhan Dinghui Chemical Co., Ltd., Wuhan, China) and euthanized by cervical dislocation after 24 h and then the right internal carotid artery was identified. Then 5 mL of blood was extracted and centrifuged. The supernatant was dispensed into two sterile tubes, sealed, and stored in a freezer at − 20 °C for analysis. Ascites and serum were collected and amylase levels and ascitic capacity were determined. Pancreata were quickly obtained and fixed in 10% formalin for observation. Portions of the pancreas were freshly treated to determine pancreatic water contents.

### RT-PCR analysis

Total RNA was extracted with TRIzol reagent (Invitrogen). The RNA concentration was measured with a Nanodrop Spectrophotometer (ND-100, Thermo, Waltham, MA, USA). cDNA was reversely transcribed from total RNA with a HiScript 1st Strand cDNA Synthesis Kit (Vazyme, Nanjing, China) according to the manufacturer’s protocol. cDNA was generated from miRNAs with a stem-loop RT-qPCR method. Quantitative real-time PCR was performed in triplicate in an ABI StepOnePlus Real-Time PCR system (Applied Biosystems, CA, USA). β-actin and U6 were adopted as endogenous controls respectively in mRNA and miRNA expression profiles. The expression levels were normalized to endogenous controls and the fold change in relative gene expression was calculated as 2^−∆∆Ct^. Primer sequences are listed in Table 1. After 10-min pre-incubation at 95 °C, PCR was performed according to the following program: 35 cycles of denaturation at 95 °C for 15 s, annealing at 60 °C for 5 s, and elongation at 72 °C for 12 s. The experiments were performed in triplicate.

**Table 1:** Primer sequences for RT-PCR

miR-181b	F-5′- ACATTCATTGCTGTCGGTGGGT-3′ R-5′-CGCTTCACGAATTTGCGTGTCA -3′	215 bp
U6	F-5′GTGCTCGCTTCGGCAGCACATATAC-3′ R-5′AAAAATATGGAACGCTCACGAATTTG-3′	237 bp
Akt mRNA	F-5′-TCACCTCTGAGACCGACACC-3′ R-5′- ACTGGCTGAGTAGGAGAACTGG-3′	174 bp
mTOR mRNA	F-5′- AGAAACTGCACGTCAGCACCA - 3′ R-5′- CCATTCCAGCCAGTCATCTTTG -3′	123 bp
Beclin1 mRNA	F-5′-GATGGTGTCTCTCGCAGATTC - 3′ R-5′-CTGTGCATTCCTCACAGAGTG -3′	247 bp
LC3-IImRNA	F-5′-GATGTCCGACTTATTCGAGAGC-3′ R-5′- TTGAGCTGTAAGCGCCTTCTA-3′	268 bp
β-actin	F-5′-GATTACTGCTCTGGCTCCTGC-3′ R-5′-GACTCATCGTACTCCTGCTTGC-3′	190 bp

### Western blot analysis

Retrieved pancreatic tissues of rats were powdered in liquid nitrogen and then lysed with a nuclear and cytoplasmic protein extract kit (Beyotime, Beijing, China). The whole proteins of pancreatic tissues were reconstituted in ice-cold RIPA buffer containing a cocktail of protease inhibitors (1:100; Sigma-Aldrich) and phenylmethanesulfonylfluoride (PMSF, 1 mM). Homogenates of pancreatic tissues were centrifuged for 15 min (12,000×g, 4 °C). Acinar cell supernatants were centrifuged for 100 min (4000×g, 4 °C) in an ultrafiltration tube (Vivaspin 20, 3000 MWCO PES, Sartorius, Germany). The concentrations of cytoplasmic, nuclear, and whole proteins were determined according to the BCA method (Pierce, Rockford, LA, USA). An aliquot of protein (80 μg) or the same proportion of concentrated supernatant was firstly separated by sodium dodecyl sulfate/polyacrylamide gel electrophoresis (SDS-PAGE Bio-Rad, Hercules, CA, USA) and then transferred to a nitrocellulose/PVDF membrane. The membrane was blocked with 5% (*w*/*v*) dry non-fat milk in Tris-buffered saline/0.05% Tween-20 (TBST) for 1 h at room temperature in a covered container. Blots were incubated with rabbit polyclonal anti-p-mTOR (1:1000), rabbit polyclonal anti-mTOR (1:1000), rabbit polyclonal anti-Beclin1 (1:200), rabbit polyclonal anti-LC3-II rabbit polyclonal (1:1000), rabbit polyclonal anti-LC3-I rabbit polyclonal (1:1000), anti-Akt antibody (1:1000), anti-p-Akt antibody (1:1000), and rat monoclonal anti-β-actin (1:1000) diluted in 5% bovine serum albumin (BSA) overnight at 4 °C. Lamin-A and β-actin were respectively used as the markers for nuclear and cytoplasmic fractions. Then the membranes were washed with TBST and incubated for 1 h at room temperature with a secondary goat anti-rabbit IgG-horseradish peroxidase (HRP) antibody (1:2000) or goat anti-rat IgG-HRP antibody (1:2000) (Santa Cruz, CA, USA) diluted in 5% (*w*/*v*) dry non-fat milk in TBST. The same protein loading of the samples was confirmed by β-actin. All western blots were determined with a densitometer.

### Immunohistochemical analysis

After antigen retrieval with Retrievagen A (Zymed Laboratories, Inc., San Francisco, CA, USA), the pancreatic tissue sections were subjected to 20-min immunostaining at 100 °C and then endogenous peroxidases were quenched with 3% H_2_O_2_ (Tianjin Jinqiang Chemical Co., Ltd.). After the sections were blocked with 2% bovine serum albumin (BSA) in phosphate-buffered saline (PBS, staining was performed at room temperature with primary anti-anti-caspase-3 and Bcl-2 (BD Pharmingen, San Jose, CA, USA) for 1 h. After washing, the sections were treated with the secondary antibody (R & D Systems, Inc.). The tissues were developed with Vectastain ABC and 3,3′-diaminobenzidine (Vector Laboratories, Inc., Burlingame, CA, USA). After staining, in each slide, five high-power fields (Magnification, 400×) were randomly selected and then the average proportion of positive expression in each field was calculated with the true color multi-functional cell image analysis management system (Rockville, MD, USA). Caspase-3 and Bcl-2-positive expressions in pancreatic tissue were measured and expressed in the form of positive units.

### Electron microscopy

After trimming pancreatic tissues to the size of 1 × 1 × 1 mm^3^, the trimmed tissues were subjected to 24-h fixation with 2.5% pentanediol and 2-hpost-fixation with 2% osmium tetroxide. The samples were respectively dehydrated according to the gradient of 50, 70, 90, and 100% dehydrated acetone and the dehydration was performed for 10 min in each concentration of dehydrated acetone for three times. Then dehydrated samples were treated at 37 °C for 24 h in the mixture of epoxy resin and pure acetone (1:1), followed by 24-h embedding at 60 °C in the mixture of Epon812 resin, dodecenylsuccinic anhydride, dimethylaminomethyl phenol, and methyl nadic anhydride. After trimming the blocks with a semi-thin glasscutter and staining with toluidine blue, the samples were observed under an optical microscopy in order to select the areas with pancreatic acinar structures. After obtaining ultrathin sections (500 Å thick) with an ultrathin microtome, the sections were stained with uranyl acetate and lead nitrate and then observed under transmission electron microscopy (Nissan HT7700; Nissan Corporation, Tokyo, Japan) to explore the changes of the pancreatic acinar autophagosomes.

### Terminal deoxynucleotidyl transferase-mediated dUTP-biotin nick-end labeling (TUNEL) assay

Apoptosis could be analyzed in the TUNEL assay (Roche Molecular Biochemicals, Mannheim, Germany). TUNEL-positive nuclei were counted in 10 random high-power fields (640× objective). The apoptotic index was calculated as a ratio of the apoptotic cell number to the total cell number in each field and expressed as a percentage. The quantification of apoptotic cells was carried out by three different observers in a blinded fashion.

### Serum endotoxin assay

Serum levels of endotoxin were determined with quantitative chromogenic endpoint Limulus Amebocyte Lysate (LAL) QCL-1000 kit (Lonza, Walkersville, MD). Firstly, 300 μL of plasma was diluted with 10 mM MgCl_2_ (Lonza) according to the ratio of 1:3 and then inactivated for 30 min at 70 °C. After the samples were further diluted to the ratio range of 1:30~ 1:40, 50 μL of the diluted sample was added into a 96-well pyrogen-free culture plate. Other procedures were performed according to the manufacturer’s instructions. Endotoxin levels (EU/mL) in the samples were obtained from a standard curve plotted with pure endotoxin standards. All the assays were performed in duplicate.

### Analysis of serum levels of D-lactate and diamine oxidase (DAO)

Serum levels of D-lactate and DAO were measured with commercial kits (Genmed, China) via spectrophotometric measurements.

### Determination of serum levels of lipase and amylase

Serum activities of lipase and amylase were determined with commercial kits in a Roche/Hitachi modular analytics system (Roche, Mannheim, Germany).

### Pancreatic water content

The changes in pancreatic weight were evaluated as the indicator of pancreatic interstitial edema. The whole pancreas was obtained and weighed. The weight of each pancreatic sample was used to estimate the water content in pancreas according to the previous method [35] and expressed as a ratio of pancreas/body weight.

### Histologic examination and scoring of pancreas

The pancreas was obtained from each rat, fixed overnight at 4 °C in 10% formalin and then embedded in paraffin. Full-length (4 μm) sections were obtained and stained with hematoxylin and eosin for histologic evaluation. According to the previous method [35], edema, hemorrhage and necrosis of the pancreas were graded into 4 levels (0 to 3).

### Pathological examination of mucosal damage

Immediately obtaining parts of distal ileum, the fixation was performed in 40 g/L phosphate buffered formaldehyde. Paraffin-embedded tissue sections (5 μm thick) were stained with hematoxylin and eosin. Mucosal damage was assessed according to the standard scale proposed by Chiu et al. [36]. Grading was classified as follows: 5 = disintegration of the lamina propria; 4 = denuded villi; 3 = massive epithelial lifting; 2 = extension of the space with epithelial lifting; 1 = development of subepithelial space at the tip of the villus; 0 = normal mucosa.

### Survival curves

The other 45 rats were divided into 3 groups: the sham operation group, SAP group and SAP plus PNS group (*n* = 15 per group) and the survival rate was calculated. The treatments were identical to those of previous experiments [3]. Observation started from PNS treatment and ended in 72 h after PNS treatment.

### Statistical analysis

In SPSS 11.0, statistical analysis was performed and the experimental data were expressed as mean ± SD. Statistical differences between two groups were evaluated by *t*-test. The analysis of linear correlation was used to evaluate the correlation between two variances and q-test of analysis of variance (ANOVA) was used to perform multiple comparisons. The survival data were analyzed with log-rank or χ2. *P* < 0.05 was considered to be significantly different.

## Results

### MiR-181b significantly down-regulated Beclin1 and LC3-II expression in AR42J cells

LC3 and Beclin-1 are the markers of autophagy [35]. To explore the effects of miR-181b on Beclin1 and LC3-II expressions, we transfected AR42J cells with MiR-181b mimics, MiR-181b mimic-negative control (NC), miR-181b inhibitor, or miR-181b inhibitor-NC. After 24-h transfection, the expression levels of Beclin1 and LC3-II were measured by Western Blotting. The increase in miR-181b expression significantly decreased Beclin1 and LC3-II expressions in the miR-181b mimics group compared to the control group and all treatment groups (*P* < 0.05) (Fig. 2). These results suggested that miR-181b might inhibit autophagy and regulate Beclin1 and LC3-II expressions.

**Fig. 2:** Effects of miR-181b on Beclin1 and LC3-II expressions in AR42J cells. MiR-181b mimics, miR-181b mimic-negative control (NC), miR-181b inhibitor, and miR-181b inhibitor-NC were transfected in AR42J cells and Beclin1 and LC3-II expressions were measured by western blotting. The data obtained from quantitative densitometry are presented as mean ± SD of three independent experiments. #*P* < 0.05 vs. control group; *P < 0.05 vs. controls and all treatment groups

### Overexpression of miR-181b inhibited pancreatic damage in the rats with SAP induced by taurocholate

To analyze the effects of overexpression of miR-181b on pancreatic damage in rats with taurocholate-induced SAP, we injected 1 × 10^9^ PFU of AdCMV-miR-181b into rats by tail intravenous administration, followed by intraperitoneal taurocholate challenge in 10 days. Histopathological examination of the pancreas of taurocholate-treated miR-181b-expressing rats revealed the markedly extenuated pancreatic damage compared with control animals (Fig. 3).

**Fig. 3:** Effects of overexpression of miR-181b on pancreas damage in the rats with SAP induced by taurocholate. Rats were injected with AdCMV-miR-181b by tail intravenous administration, followed by intraperitoneal taurocholate challenge in 10 days. Histopathological examination of pancreas tissues was performed. **a** Images of hematoxylin and eosin-stained pancreas sections from SO group, SAP group and miR-181b-expressing group. (Magnification, 400×; Scale Bar: 50 μm). **b** Pancreas damage scores. Pancreas damage scores are expressed as mean ± SD of three replicates. ##*P* < 0.01 vs. the model group; **P < 0.01 vs. the control group

### Overexpression of miR-181b decreased Beclin1 and LC3-II expressions in rats with SAP induced by taurocholate

To analyze the effects of overexpression of miR-181b on Beclin1 and LC3-II expression in rats with taurocholate-induced acute pancreatitis, we performed western blotting on pancreatic tissue samples. As shown in Fig. 4, taurocholate-induced SAP tissues in SAP/miR-181b group and SAP group showed the significantly increased Beclin1 and LC3-II expressions compared to the SO group and SO/miR-181b group (*P* < 0.05). However, overexpression of miR-181b in rats with taurocholate-induced AP (the SAP/miR-181b group) resulted in the decreased Beclin1 and LC3-II expressions compared to the rats induced by taurocholate (SAP group) (*P* < 0.05).

**Fig. 4:** Effects of overexpression of miR-181b on LC3-II and Beclin1 expressions in rats with SAP induced by taurocholate. The expressions of LC3-II and Beclin1 in the SO group, SO miR-181b group, SAP group and SAP miR-181b group were measured via Western Blot analysis. Each value represents mean ± SD of three independent experiments. ##*P* < 0.01, *#P* < 0.05 vs. the control group; **P < 0.01, *P < 0.05 vs. the normal control group

### Effects of PNS on the expressions of miR-181b, mTOR, Akt, Beclin1 and LC3-II in taurocholate-induced pancreas tissue

We evaluated the effects of PNS treatment on SAP rats by examining the expressions of miR-181b, mTOR, Akt, Beclin1 and LC3-II in taurocholate-induced pancreas tissue by RT-PCR and Western Blotting. In taurocholate-induced rats, the mRNA and proteins of miR-181 and mTOR were significantly decreased (*P* < 0.05) and Akt, Beclin1 and LC3-II expressions were significantly upregulated compared to the control group (*P* < 0.05). After PNS treatment, the expressions of miR-181 and mTOR were markedly enhanced (*P* < 0.05), whereas Akt, Beclin1, and LC3-II expressions were significantly lower compared to the SAP group (*P* < 0.05). The changes suggested that PNS could suppress the expressions of Akt, Beclin1 and LC3-II, and upregulate miR-181b and mTOR expressions (Figs. 5–6).

**Fig. 5:** Effects of PNS on the expressions of miR-181b, mTOR, Akt, Beclin1, and LC3-II mRNA in pancreas tissues from the rats with SAP induced by **taurocholate. a** RT-PCR results of miR-181b, LC3-II, mTOR, Akt, Beclin1, and mRNA in the SO group, SAP group and PNS treatment group. **b** Statistical analysis of densitometric data of mRNA levels from (A). Each value represents mean ± SD of three independent experiments. ##*P* < 0.01, #*P* < 0.05 vs. the SAP group; **P < 0.01, *P < 0.05 vs. sham operation group

**Fig. 6:** Effects of PNS on the protein expressions of p-mTOR, p-Akt, Beclin1 and LC3-II in taurocholate-induced rat pancreas tissues. a Representative western blots of p-mTOR, p-Akt, Beclin1, and LC3-II protein expressions in all three groups. **b** Statistical analysis of densitometric data of the data from (A). Data are expressed as mean ± SD of three experiments. #*P* < 0.01, ##*P* < 0.01 vs. the SAP group; **P < 0.01, *P < 0.05 vs. the sham operation group

### Effects of PNS on pancreatic autophagy in taurocholate-induced rat pancreas tissues

The formation of autophagosomes is a pivotal process in autophagy. To explore the effect of PNS on autophagy in SAP, the ultrastructures of pancreatic cells from the three treatment groups were observed under the electron microscopy. Phagophores, autophagosomes and autolysosomes were increased in the taurocholate-treated group and decreased in the PNS treatment group (Fig. 7). These observations suggested that PNS inhibited pancreatic autophagy in taurocholate-induced rat pancreas tissues.

**Fig. 7:** Autophagosome formation detected in pancreatic tissues. Autophagosomes in representative transmission electron microscopy images from three treatment groups are indicated with arrows. Six fields were randomly selected in each slice and autophagosomes were calculated as average positive rate. (Original magnification, 15,000×; Scale Bar: 2 μm). Data are expressed as mean ± SD of three experiments. #*P* < 0.05 vs. the SAP group; *P < 0.05 vs. the sham operation group

### PNS treatment increased caspase-3 expression in pancreas tissues with taurocholate-induced SAP

The effects of PNS treatment on apoptosis in the SAP model was explored by evaluating Bcl-2 and caspase-3 expressions in pancreas tissues via immunohistochemistry. The expressions of Caspase-3 and Bcl-2 were significantly up-regulated in pancreas tissues from the rats with taurocholate-induced SAP (Fig. 8). However, administration of PNS further significantly decreased Bcl-2 expression and increased Caspase-3 expression in taurocholate-induced SAP rats. These results demonstrated that PNS significantly activated Caspase-3 expression and enhanced Bcl-2 expression in SAP model rats.

**Fig. 8:** Effect of PNS on the expression of caspase-3 and Bcl-2 in pancreas tissues from rats with taurocholate-induced SAP. The levels of Caspase-3 and Blc-2 were assayed by immunohistochemistry in all the treatment groups (Scale Bars: 20 μm). Data are expressed as mean ± SD of three experiments. #*P* < 0.01, ##*P* < 0.01 vs. the control group; **P < 0.01, *P < 0.05 vs. the sham operation group

### PNS treatment increased the apoptotic rate of pancreatic cells in taurocholate-exposed SAP rats

The effects of PNS treatment on the apoptosis of pancreatic cells from taurocholate-exposed SAP rats were explored via TUNEL assays. In the rats exposed to taurocholate, the apoptotic rate of pancreatic cells was significantly higher than that in the control group (Fig. 9). Notably, compared to the taurocholate group, the PNS treatment group exhibited a significantly increased apoptotic rate of pancreatic cells (*P* < 0.05). The differences suggested that PNS increased the apoptosis in pancreatic cells in the SAP model rats.

**Fig. 9:** Effects of PNS treatment on the apoptosis of pancreatic cells in the rats with taurocholate-induced SAP. TUNEL analysis was performed in the three treatment groups. TUNEL images showed the apoptosis of pancreatic cells in rats in 24 h after PNS administration (Magnification, 200 ×; Scale Bars: 50 μm)

### Effects of PNS treatment on the ratio of pancreas to body weight and serum amylase activity

In pancreatitis assessment, pancreatic edema is one of the key factors [29, 37]. After injecting 5% sodium taurocholate into the biliary-pancreatic duct of rats in our model, the pancreas/body weight ratio was significantly increased (Fig. 10). Furthermore, serum amylase activity in the SAP rats was significantly increased. Notably, PNS treatment largely decreased the ratio of pancreas to body weight as well as serum amylase activity, showing a positive effect on pancreatic injury and edema.

**Fig. 10:** Effects of PNS treatment on the ratio of pancreas to body weight as well as serum amylase activity. The ratio of pancreas to body weight as well as serum amylase activity was determined in all the three groups. Data represent mean ± SD of three experiments. * *P* < 0.05 and **P < 0.01 compared with the control group; #*P* < 0.05 and ##*P* < 0.01 compared with the taurocholate group

### Effects of PNS treatment on plasma D-lactic acid, DAO and endotoxin in rats with taurocholate-induced AP

Previous studies indicated that intestinal barrier injury might lead to the multiple organ dysfunction syndrome [38]. We examined plasma D-lactic acid and DAO with the two markers indicating intestinal barrier dysfunction caused by SAP. We determined the two markers by ELISA and serum endotoxin (Fig. 11). In the SAP model group, the plasma DAO, D-lactic acid, and serum endotoxin were significantly increased compared to the control group. Notably, compared with the SAP group, the PNS group exhibited the significantly decreased plasma D-lactic acid, DAO and endotoxin (*P* < 0.05). Our results showed that administration of PNS significantly reduced plasma D-lactic acid, endotoxin, and DAO in SAP rats.

**Fig. 11:** Effects of administration of PNS on the plasma D-lactic acid, diamine oxidase and endotoxin in rats with taurocholate-induced SAP. Plasma D-lactic acid, diamine oxidase and endotoxin in the three groups of rats were evaluated. Data are expressed as mean ± SD of three experiments. ##*P* < 0.01 and #*P* < 0.05 vs the taurocholate group; **P < 0.01 and *P < 0.05 vs the control group

### Effects of PNS on pancreatic and ileal histology

In order to evaluate the effects of PNS on local pancreatic and ileal injury, the morphology of the pancreas in the rats of all the three groups was observed (Fig. 12). The SAP group exhibited the severe edema and the high destruction degree of histoarchitecture of acini cells and pancreatic pathological scores in the SAP group were significantly increased compared to the model group. After establishing SAP models, villi and crypt structures were damaged to some extent and hair became thinner and shorter. Heavy inflammatory cell infiltration in the intrinsic membrane was observed and lymphatic dilatation and edema occurred. In the PNS treatment group, the injury to ileal and pancreatic tissues was attenuated and pancreatic and ileal injury scores were significantly reduced. These data suggested that PNS treatment attenuated the injury to pancreatic and ileal tissues.

**Fig. 12:** Histopathological changes of pancreatic and ileal tissues in rats upon PNS treatment. **a** Histopathological changes in pancreatic and ileal tissues (Magnification: 200×; Scale Bar: 50 μm). **b** Statistical analysis of pancreatic and ileal pathological scores in rats. Pancreatic and ileal injury scores were expressed as mean ± SD from triplicate experiments. ##*P* < 0.01 vs. the control group; **P < 0.01 vs. the sham operation group

### Effects of PNS on the survival rate of rats

The survival rate of the rats with taurocholate-induced SAP was significantly decreased compared to the control group. The decreasing trend in the survival rate induced by taurocholate-induced SAP was significantly attenuated by the pre-treatment with PNS compared to the untreated taurocholate-induced SAP group (Fig. 13).

**Fig. 13:** Survival curve. SAP group is the group treated with taurocholate; SAP + PNS group is the group firstly treated with taurocholate and then treated with PNS. #*P* < 0.05 vs. SAP group; * *P* < 0.05 vs. sham operation group. SAP, severe acute pancreatitis. h, hour

## Discussion

AP is a clinical challenge because the pathogenesis of AP remains elusive and its specific treatment method is not available [39]. We examined the potential effectiveness of PNS against AP and found that PNS markedly decreased the pancreas/body weight ratio as well as serum amylase activity, significantly reduced intestinal barrier injury, and extenuated pancreatic injury. These effects may be mediated by inducing miR-181b and mTOR expressions in pancreas and subsequently reducing autophagosome formation, which is important for initiating pancreatitis [40–42].

Autophagy in acinar cells largely determines the development of pancreatitis. Impaired autophagic influx is a key mechanism of intra-acinar trypsin activation and pancreatitis [40, 42, 43]. The rats with the deficiency in the formation of autophagosomes are resistant to AP [44], indicating that the formed autophagosomes is also important in the development of pancreatitis. In the study, taurocholate-induced autophagosome formation was diminished upon PNS treatment in SAP rats (Fig. 8), confirming that the protection effect of PNS on taurocholate-induced pancreatitis was realized by inhibiting the formed autophagosomes. In addition, PNS treatment extenuated SAP by attenuating autophagy activation via increasing the mTOR/Akt pathway. It is another possible mechanism of the protection effect of PNS.

Some signaling pathways are involved in the regulation of autophagy [45]. The PI3K/Akt pathway is an important anti-apoptosis/proliferation signaling pathway in key cellular functions [45]. Activated Akt is a downstream effector of PI3K and PI3K regulates the autophagy function via upstream Beclin1 and mTOR and comprises a PI3K-Beclin1-mTOR regulatory network of autophagy [46]. This “double-edged sword” effect was observed. A slight increase in autophagy inhibited apoptosis and promoted cell survival during the SAP period. On the contrary, an abnormal increase in autophagy aggravated pancreas injury during the SAP period [47]. It had been reported that the activation of the PI3K/Akt signaling pathway could suppress apoptosis and excessive autophagy. Lupia et al. [48] knocked out the PI3K gamma gene in rats to establish an AP model and found that the injury and necrosis of pancreatic acinar cells were markedly decreased compared with wild-type rats. Jia and Sun [49] found that after the PI3K gamma gene in rats was knocked out, AP was induced and the number of vacuoles in pancreatic acinar cells, the number of LC3-II particles, and activity of trypsinogen were significantly decreased, suggesting that PI3K enhanced autophagy of pancreatic acinar cells, promoted activation of plasminogen, and further accelerated cell death.

Autophagosomes have two markers: LC3-II and Beclin1, which are up-regulated in the reperfusion period [49]. Our data suggested that taurocholate-induced AP decreased the activity of miR-181b, stimulated the activity of the PI3K/Akt signaling pathway, attenuated the activity of mTOR pathway, enhanced Beclin1 and LC3-II expression, and increased pancreatic cell autophagy, pancreatic cell apoptosis, and taurocholate-induced AP. However, the administration of PNS increased the activity of mTOR and miR-181b, inhibited Beclin1 and LC3-II expression, decreased pancreatic cell autophagy, enhanced pancreatic cell apoptosis, and ameliorated taurocholate-induced AP. Bcl-2 played a key role in the inhibition of the stimulatory Beclin-1 pathway [50]. In the study, the administration of PNS enhanced the reduction of Bcl-2 induced by SAP, attenuated Beclin-1 expression, decreased pancreatic cell autophagy and further ameliorated taurocholate-induced AP.

Recent studies suggested that apoptosis could be a beneficial reaction to AP [51, 52]. Caspase-3 is involved in various forms of apoptosis [53] and dispensable in some forms of apoptosis [54]. In podocytes, puromycin aminonucleoside activated caspase-3 [55]. Furthermore, the activated caspase-3 is caused by Bcl-2 insufficiency [56]. In the study, taurocholate-induced AP attenuated caspase-3 and increased Bcl-2. We found that PNS increased apoptosis and that Bcl-2 and other proteins in the caspase pathway might be involved in PNS-induced increase of apoptosis. In addition, caspase-3 activity was increased in PNS-treated taurocholate-induced AP. We proved that the increase of apoptosis by PNS induction markedly improved taurocholate-induced pancreatic injury.

In the study, miR-181b expression was significantly down-regulated in the AP model. We hypothesized that miR-181b played an important role in the development of AP. Furthermore, we transfected AR42J cells with miR-181b mimics and indicated that Beclin1 and LC3-II expressions were significantly decreased compared with the control group and all treatment groups (*P* < 0.05). To further investigate the effects of miR-181b on taurocholate induced-AP, we injected AdCMV-miR-181b into rats by tail intravenous administration, followed by intraperitoneal taurocholate challenge in 10 days, and found that the overexpression of miR-181b inhibited Beclin1 and LC3-II expression, reduced autophagy, and inhibited pancreatic damage in rats with taurocholate-induced AP. The study results suggested that overexpression of miR-181b protected taurocholate-induced AP by inhibiting autophagy apoptosis and promoting autophagy via regulating Beclin1 and LC3-II expression. In the SAP model, we found that taurocholate-induced AP decreased the activity of miR-181b and increased the activity of the mTOR/Akt pathway. Therefore, the downregulation of miR-181b might affect pancreas tissues in AP by regulating the activity of the mTOR/Akt pathway. Moreover, PNS increased the activity of miR-181b, stimulated the activity of the mTOR/Akt pathway, decreased LC3-II and Beclin1 expressions, reduced the number of phagophores, autophagosomes and autolysosomes, reduced autophagy, and ameliorated taurocholate-induced AP.

MiR-181a and miR-181b of the miR-181 family are tumor suppressors for inducing apoptosis [57]. MiR-181 induced apoptosis in astrocytes by targeting multiple members of the Bcl-2 family [58]. Moreover, miR-181 significantly enhanced drug-induced apoptosis in cancer cells by targeting multiple anti-apoptosis genes, such as Bcl-2 [57, 58]. In the study, administration of PNS significantly decreased Blc-2 expression and increased caspase-3 expression by increasing miR-181b expression, promoting pancreatic acinar cell apoptosis, and reducing taurocholate-induced pancreatic injury.

Intestinal mucosa injury is mainly responsible for the accelerated aggravation of SAP and can aggravate SAP. Our results showed that administration of PNS attenuated intestinal mucosa injury, and resulted in a reduction of endotoxemia, thus ameliorating SAP. Furthermore, as indicated by the two markers (D-lactate and DAO), PNS could decrease DAO and D-lactate in taurocholate-induced SAP rats. Therefore, the administration of PNS could largely improve the intestinal barrier function and reduce the intestinal mucosal damage caused by SAP.

## Conclusions

PNS showed a protective effect on taurocholate-induced SAP and exerted a therapeutic effect through upregulating the miR-181b expression, decreasing the activity of mTOR/Akt pathway, attenuating Beclin1 and LC3-II expressions, enhancing the activity of caspase-3 pathway, increasing pancreatic cell apoptosis, reducing autophagy, ameliorating the impaired intestinal mucosal barrier, attenuating taurocholate-induced pancreatic damage, and increasing the survival rate in taurocholate-induced SAP rats. Our findings provided the basis for the clinical application of PNS in the treatment of AP.

## Abbreviations

Akt: Protein kinase B
Beclin1: Myosin-like Bcl2 interacting protein
LC3-II: Microtubule-associated protein II light chain 3
MiRNA: micrornas
MTOR: Mammalian target of rapamycin
PI3K: Phosphatidylinositol-3-kinase
SAP: Severe acute pancreatitis
